# Comparison of Five Triage Tools for Identifying Mortality Risk and Injury Severity of Multiple Trauma Patients Admitted to the Emergency Department in the Daytime and Nighttime: A Retrospective Study

This article has been retracted.

**DOI:** 10.1155/2022/9368920

**Published:** 2022-02-25

**Authors:** Youguo Ying, Boli Huang, Yan Zhu, Xiaobin Jiang, Jinxiu Dong, Yanfen Ding, Lei Wang, Huimin Yuan, Ping Jiang

**Affiliations:** ^1^Emergency Department 1, Shanghai Ninth People's Hospital, Shanghai Jiao Tong University School of Medicine, Shanghai, China; ^2^Department of Nursing, Shanghai Ninth People's Hospital, Shanghai Jiao Tong University School of Medicine, Shanghai, China; ^3^Nursing Management Research Center of China Hospital Development Institute, Shanghai Jiao Tong University, Shanghai, China; ^4^Independent Researcher, Tokyo, Japan

## Abstract

Effective triage tools are indispensable for doctors to make a prompt decision for the treatment of multiple trauma patients in emergency departments (EDs). The Modified Early Warning Score (MEWS), National Early Warning Score (NEWS), standardized early warning score (SEWS), Modified Rapid Emergency Medicine Score (mREMS), and Revised Trauma Score (RTS) are five common triage tools proposed for trauma management. However, few studies have compared these tools in a multiple trauma cohort and investigated the influence of nighttime admission on the performance of these tools. This retrospective study was aimed at evaluating and comparing the performance of MEWS, NEWS, SEWS, mREMS, and RTS for identifying the mortality risk and trauma severity of patients with multiple trauma admitted to the ED during the daytime and nighttime. Retrospective data were collected from the medical records of patients with multiple trauma admitted in the daytime or nighttime to calculate scores for each triage tool. Logistic regression analysis was conducted on each triage tool for identifying in-hospital mortality and severe trauma (injury severity score > 15) in the daytime and nighttime. The performance of the tools was evaluated and compared by calculating area under the receiver operating characteristic curve (AUROC) of the retrospective logistic model of each tool. We collected data for 1,818 admissions, including 1,070 daytime and 748 nighttime admissions. A comparison of performance for identifying in-hospital mortality between daytime and nighttime yielded the following results (AUROC): MEWS (0.95 vs. 0.93, *p* = 0.384), NEWS (0.95 vs. 0.94, *p* = 0.708), SEWS (0.95 vs. 0.94, *p* = 0.683), mREMS (0.94 vs. 0.92, *p* = 0.286), and RTS (0.93 vs. 0.93, *p* = 0.87). Similarly, a comparison of performance for identifying trauma severity between daytime and nighttime yielded the following results (AUROC): MEWS (0.78 vs. 0.78, *p* = 0.95), NEWS (0.8 vs. 0.8, *p* = 0.885), SEWS (0.78 vs. 0.78, *p* = 0.818), mREMS (0.75 vs. 0.69, *p* = 0.019), and RTS (0.75 vs. 0.74, *p* = 0.619). All five scores are excellent triage tools (AUROC ≥ 0.9) for identifying in-hospital mortality for both daytime and nighttime admissions. However, they have only moderate effectiveness (AUROC < 0.9) at identifying severe trauma. The NEWS is the best triage tool for identifying severe trauma for both daytime and nighttime admissions. The MEWS, NEWS, SEWS, and RTS exhibited no significant differences in performance for identifying in-hospital mortality or severe trauma during the daytime or nighttime. However, the mREMS was better at identifying severe trauma during the daytime.

## 1. Introduction

Multiple trauma is fatal due to sequelae such as traumatic shock, respiratory failure, or multiple organ dysfunction syndrome, leading to a high risk of mortality among patients. In particular, approximately 4,000 people die from multiple trauma each year in China [1, 2]. Thus, effective triage tools are indispensable for physicians to rapidly identify the risk of mortality in patients presenting to the emergency department (ED) with multiple trauma.

There are various trauma triage tools, such as National Early Warning Score (NEWS) [3], Modified Early Warning Score (MEWS) [4], standardized early warning score (SEWS) [5], Modified Rapid Emergency Medicine Score (mREMS) [6], and Revised Trauma Score (RTS) [7], that have been widely used in EDs because they are easy and convenient to memorize, utilize, and assess. Compared with anatomical-based triage tools (e.g., injury severity score (ISS) [8] and Abbreviated Injury Scale (AIS) [9]), these tools do not require specialized knowledge for assessing injury severity or calculating scores. In addition, the five scoring systems include fewer variables than anatomical systems, and the included variables can be measured and calculated rapidly without specialized medical equipment. These five scoring systems include only 4-6 variables, in contrast to more complicated systems such as the Acute Physiology, Age, and Chronic Health Evaluation (APACHE) III score [10], which includes 17 variables. Thus, these five common triage tools have been widely used for risk-stratification measurement [11, 12], mortality risk prediction [5, 13–16], need of intensive care unit (ICU) admission [17–19], and trauma severity assessment [20, 21].

However, few previous studies have compared the performance of these five triage tools in consideration of daytime and nighttime admission based on data from a multiple trauma cohort. Those previous studies mainly compared the performance of triage tools for identifying mortality risk among patients with coronavirus disease 2019 [22–24], those with splenic abscess [25], those who were elderly [26, 27], those admitted to the general ED [28–31], and patients with trauma [32–35], without considering the patient admission time. However, Hirose et al. [36] reported that mortality is significantly lower among patients admitted to the ED during the daytime than among those admitted during the nighttime. Barbosa et al. [37] also reported that nighttime admission was associated with surgical mortality in patients with trauma. Hence, it is necessary to investigate whether time of day affects the performance of these triage tools.

Therefore, the present retrospective study was aimed at evaluating and comparing the performance of the NEWS, MEWS, SEWS, mREMS, and RTS in identifying the in-hospital mortality and trauma severity of multiple trauma patients admitted to the ED during the daytime or nighttime. Logistic regression analysis was conducted on a retrospective multiple trauma cohort dataset to investigate the correlation of each tool with in-hospital mortality and trauma severity. The area under the receiver operating characteristic (AUROC) of the logistic regression result of each tool was calculated to evaluate the performance. We assumed a triage tool whose AUROC ≥ 0.9 as an excellent tool with high discrimination ability for identifying patient outcome.

## 2. Materials and Methods

### 2.1. Ethical Statement

This retrospective study was approved by the research ethics committee of Shanghai Ninth People's Hospital (approval number: 2020-T368-2), which waived the requirement for informed consent due to the nature of the study.

### 2.2. Data Collection

Data for this retrospective study were collected from the medical records of patients with multiple trauma admitted to the ED of an urban hospital between May 2014 and April 2020. Shanghai Ninth People's Hospital has the second largest emergency center in Shanghai, with 50 beds for patient admission. Annually, it admits approximately 20,000 trauma patients, among whom 3,000 are multiple trauma patients. ED doctors measured the vital signs and made decisions for medical examinations and trauma triage for all the patients immediately once they were admitted. Generally, ED doctors work on a rotational shift schedule such that if they work during the daytime on one day, they will work during the nighttime the next few days.

The medical records of multiple trauma patient cohort were picked out among all ED patients through the review of the medical examination results (e.g., computed tomography (CT)) by a trauma specialist. Patients were identified as having multiple trauma if they suffered from injury to two or more bodily regions, with at least one injury being potentially life-threatening [38].

The extracted medical record data of the multiple trauma patient cohort was further filtered based on the following inclusion criteria. We included only adult patients (age ⩾16), based on the design of the scoring systems (e.g., MEWS). Patients with incomplete medical records (e.g., all variables for score calculation are missing) were excluded because their data may have biased the results and it would have been difficult to perform data imputation. Furthermore, we excluded patients with a history of prior injury, infection, or organ dysfunction that may have made it difficult to determine whether outcomes (e.g., mortality) were caused by multiple trauma.

The included cohort was divided into daytime and nighttime populations based on the time of admission. There are no standard criteria for determining the boundary between daytime and nighttime because sunshine durations are different in different regions of the world. We empirically defined daytime as 8:01 am to 17:59 pm and nighttime as 18:00 pm to 8:00 am based on local daytime duration and the hospital's official working hours (http://www.9hospital.com.cn). The daytime and nighttime cohorts were divided into survival and nonsurvival groups according to in-hospital mortality records. In-hospital mortality cohort also included all those who died within 90 days. The same two cohorts were divided into minor and severe trauma groups. Severe trauma was defined as an ISS > 15, in accordance with previous definitions [39].

For each included case, we collected the variables required to calculate the score of the five triage tools (Table 1). Systolic blood pressure (SBP) and respiratory rate (RR) were collected because all five triage tools use them to calculate the score. Heart rate (HR), temperature (*T*), oxygen saturation (SaO_2_), and the Alert, Verbal, Pain, and Unresponsive score (AVPU) [4] were further collected to calculate the score of MEWS [4], SEWS [5], and NEMS [3]. Glasgow Coma Scale (GCS) score was collected to calculate the scores of mREMS [6] and RTS [7]. AVPU and GCS are both assessments of consciousness level, and AVPU can be derived from GCS as follows: 14–15 for A, 9–13 for V, 4–8 for P, and 3 for U [4]. Data on age was also acquired for assessing mREMS. In addition to the variables related to the triage tools, we also collected details on sex, length of stay (LOS) in the hospital, and trauma mechanism.

### 2.3. Statistical Analysis

Statistical analysis was performed to summarize the data characteristics of the included cohort. Multivariate imputation by chained equations (MICE) was performed to impute missing values. Cases were directly excluded without imputation if all variables required to calculate the score of a tool (Table 1) were missing because it would be difficult to impute. Normally distributed numerical variables are expressed as means (standard variation (std)) and were compared using *t*-tests. Nonnormally distributed numerical variables are expressed as medians (interquartile ranges (IQRS)) and were compared using the Wilcoxon-Mann-Whitney test. Categorical variables are expressed as frequencies and were compared using Pearson's chi-square test.

The scores of each triage tool of the included cohort were calculated based on Table 1. To compare the performance of the tools, logistic regression analysis was performed on the daytime and nighttime admission cohorts, respectively, in order to investigate the correlation of the score of each tool with in-hospital mortality and trauma severity. AUROC of the logistic regression model was calculated to evaluate the performance (predictive validity) of identifying in-hospital mortality and severe trauma for the five triage tools. For clinical application, cut-offs are important for doctors or nurses to make triage decisions. Hence, the optimal (Opt) cut-off point of the receiver operating characteristic curve of each triage tool was calculated, and sensitivity (Sen) and specificity (Sp) at the optimal cut-off were evaluated. All statistical analyses were conducted using R, version 4.0.2 (R foundation for Statistical Computing, Vienna, Austria).

## 3. Results

### 3.1. Data Characteristics

As shown in Figure 1, the cohort included 1,818 eligible patients with multiple trauma, comprising 1,070 daytime admissions and 748 nighttime admissions. All patients arrived in cars or walked into the ED by themselves. Seventy-one patients (3.91%) had missing values that were imputed by MICE. Among these 71 patients, 15 had missing values for only 1 variable (*T*, SBP, or SaO_2_), 5 had missing values for 2 variables (SBP and SaO_2_ or RR and SaO_2_), 14 had missing values for 3 variables (RR, SBP, and SaO_2_ or HR, SBP, and SaO_2_), and 37 had missing values for 4 variables (HR, RR, SBP, and SaO_2_).

The daytime survival and nonsurvival groups included 917 and 153 patients, while the nighttime survival and nonsurvival groups included 651 and 97 patients, respectively. The characteristics of the survival and nonsurvival groups for patients admitted during the daytime and nighttime are presented in Table 2. The daytime minor and severe trauma groups included 703 and 367 patients, while the nighttime minor and severe trauma groups included 495 and 253 patients, respectively. The characteristics of the minor and severe trauma groups are shown in Table 3. The main trauma mechanism (cause of injury) in all groups was traffic accidents and tumble injury. As expected, those that survived had longer length of stay (LOS) in the hospital than those that did not.

### 3.2. Performance of Identifying In-Hospital Mortality for Daytime and Nighttime Admissions

As shown in Figure 2 and Table 4, for all five scores, the AUROC values for identifying in-hospital mortality were ≥0.9 for patients admitted during either the daytime or nighttime. Among all scores, the NEWS had the highest sensitivity during the daytime at its optimal cut-off, while the NEWS and SEWS had the highest sensitivity during the nighttime. *p* values for the comparison of ROCs for daytime and nighttime were all >0.05, indicating that there were no significant differences in the ability of the scores to identify mortality during either the daytime or nighttime.

### 3.3. Performance of Identifying Trauma Severity for Daytime and Nighttime Admissions

As shown in Figure 3 and Table 5, AUROC values for identifying severe trauma were lower than those for identifying in-hospital mortality for all five scores (Table 4), during both daytime and nighttime. Among all scores, the NEWS had the highest AUROC and sensitivity for both daytime and nighttime admissions. There were no significant differences in the ability to identify severe trauma during the daytime and nighttime for the MEWS, NEWS, SEWS, or RTS. However, mREMS performance was better during the daytime than during the nighttime (AUROC 0.75 vs. 0.69, *p* = 0.019).

## 4. Discussion

This retrospective study was aimed at comparing the performance of five common trauma triage tools for identifying in-hospital mortality and severe trauma in patients admitted to the ED with multiple trauma during the daytime and nighttime.

For identifying in-hospital mortality, our findings indicated that the MEWS, NEWS, SEWS, REM, and RTS are all excellent triage tools (AUROC ≥ 0.9) for both daytime and nighttime admissions. Indeed, we observed no significant differences (*p* value > 0.05) in the performances of each triage tool between daytime and nighttime admissions (Table 4). This result is in accordance with a previous finding showing that admission time may not influence in-hospital mortality. Dybda et al. [40] reported that nighttime admission was not a significant predictor of mortality in patients with severe trauma. The same result was derived from a larger cohort study in the UK by Metcalfe et al. [41]. However, several studies have demonstrated associations between the daytime/nighttime scoring system variables (Table 1) and patient outcomes. Fagard et al. [42] reported that nighttime SBP is a better predictor of mortality than daytime SBP in patients with hypertension. Hirose et al. [36] further reported that daytime/nighttime admission is associated with mortality in adult patients. Yue et al. [43] argued that GCS is more important for determining the need for ICU admission during the daytime than during the nighttime. In addition, Palatini et al. [44] showed that nighttime HR is a better predictor of cardiovascular events in patients with hypertension than daytime HR. Although these findings are in contrast to ours, these studies did not include patients with multiple trauma.

Furthermore, by comparing the specific AUROC values of the tools, we found that there was only a small difference in the AUROC values between the triage tools for identifying in-hospital mortality for either daytime or nighttime. This result is partly in accordance with that reported by a previous study using another cohort but without considering admission time. Hu et al. [22] reported that the SEWS and NEWS were superior to the MEWS (AUROC: 0.84, 0.81 vs. 0.67) for predicting mortality in patients with coronavirus disease 2019. Mitsunaga et al. [26] found no significant difference between the NEWS and MEWS (AUROC: 0.68 vs. 0.65) in prehospital settings, whereas the NEWS performed better than the MEWS(AUROC: 0.79 vs. 0.72) in ED settings, although the majority of the cohort was composed of nontrauma cases. Lee et al. [28] further demonstrated that the NEWS is superior to the MEWS and REMS (AUROC: 0.81 vs. 0.78, 0.75) for predicting in-hospital mortality within 30 days. Similar AUROC values for the ability of the REMS and RTS (0.91 vs. 0.89) to predict in-hospital mortality in patients with trauma have been reported [33]. Cattermole et al. [29] reported that the MEWS, REMS, and RTS exhibit similar performance (AUROC: 0.75 vs. 0.77 vs. 0.77) in predicting 30-day in-hospital mortality. This study makes a significant contribution to the literature because we compared AUROC values of triage tools based on multiple cohorts considering the admission time, which has not been reported previously.

To the best of our knowledge, this is the first study to compare the predictive validity of scoring systems for identifying severe trauma in consideration of admission time. Our results showed that the mREMS performed better for daytime admissions than for nighttime admissions, while no significant differences were observed for the MEWS, NEWS, SEWS, or RTS (Table 5). The NEWS outperformed other scores for identifying severe trauma for both daytime and nighttime admissions. Hence, attention should be paid when using the mREMS during the nighttime; otherwise, a more reliable tool (such as the NEWS) for identifying severe trauma should be chosen.

In addition, we observed that all five scoring systems were better at identifying in-hospital mortality than severe trauma for both daytime and nighttime admissions. This result agrees with the findings of a previous study [20], which showed that scoring systems were only moderately effective as triage tools for trauma severity. This may be because the scoring systems were designed only for assessing mortality rather than trauma severity. One way to improve performance for identifying severe trauma is to redesign the range of variables in the scoring system. Jeong et al. [45] reported improvements in the ability of the RTS to predict in-hospital mortality when the SBP range was revised. The same concept can also be used to improve the ability to predict trauma severity. Alternatively, performance can be improved by adding variables associated with trauma severity to the scoring system. Jiang [21] incorporated an abdominal injury severity variable into the traditional MEWS, which improved the AUROC for identifying severe trauma.

Based on the results of this study, we recommended the clinical application of the triage tools in the ED. As can be seen in Table 4, the NEWS had higher AUROC values and sensitivity; thus, it should be preferentially chosen to identify mortality risk during daytime and nighttime. Patients with NEWS > 4 at daytime or NEWS > 5 at nighttime are supposed to have high mortality risk; hence, they should be properly triaged so that further assessment and treatment can be undertaken. On the other hand, as seen in Table 5, the NEWS should also be preferentially used for identifying severe trauma during both daytime and nighttime. As severe trauma may lead to acute deterioration of the patient's condition, the NEWS can be used to determine the need for and frequency of monitoring in admitted patients.

The present study had some limitations, including its retrospective, single-center design. More samples from multiple local urban hospitals are required to further validate our findings. In addition, daytime and nighttime durations may vary due to the location of the hospital. Thus, it remains necessary to compare findings among urban hospitals in various cities or countries. Furthermore, although multiple trauma was assessed by a trauma specialist based on medical records and CT findings, the diagnosis was subjective and was not made in real time. In addition, the medical records were documented by different ED staff within a short time frame, which may have led to variations. In addition, other factors, such as different types of trauma and orthopedic fractures [46], which were not included in the triage tool, may also be associated with in-hospital mortality. In future studies, we will also include those factors to further improve the performance of the triage tool.

## 5. Conclusions

The MEWS, NEWS, SEWS, REM, and RTS are all excellent triage tools for identifying in-hospital mortality for both daytime and nighttime admissions. Our analysis revealed no significant differences in the ability of these five systems to predict in-hospital mortality between daytime and nighttime admissions. However, the MEWS, NEWS, SEWS, REM, and RTS exhibit only a moderate ability to identify severe trauma. Our findings indicate that the NEWS is the best triage tool with the highest AUROC and sensitivity for identifying severe trauma for both daytime and nighttime admissions. While there were no significant differences in the ability of the MEWS, NEWS, SEWS, and RTS to identify severe trauma between daytime and nighttime, the mREMS performed better during the daytime than during the nighttime.

## Figures and Tables

**Figure 1:** Composition of included cohort.

**Figure 2:** ROC curves for identifying in-hospital mortality among patients with multiple trauma admitted during the daytime and nighttime for five triage scores.

**Figure 3:** ROC curves for identifying severe trauma in patients with multiple trauma admitted during daytime and nighttime for five triage scores.

**(a):** 

MEWS							
Variable	3	2	1	0	1	2	3
SBP (mmHg)	<70	70–80	81-100	101-199		≥200	
HR (beats/min)		<40	40-50	51-100	101-110	111-129	≥130
RR (cycles/min)		<9		9-14	15-20	21-29	≥30
*T* (°C)		<35		35–38.4		≥38.5	
AVPU				A	V	P	U

**(b):** 

SEWS							
Variable	3	2	1	0	1	2	3
SBP (mmHg)	<70	70–79	80-99	100-199		≥200	
HR (beats/min)	<30	30-39	40-49	50-99	100-109	110-129	≥130
RR (cycles/min)	<9			9-20	21-30	31-35	≥36
*T* (°C)	<34	34-34.9	35-35.9	36–37.9	38-38.9	≥39	
SaO_2_ (%)	<85	85-89	90-92	≥93			
AVPU				A	V	P	U

**(c):** 

NEWS							
Variable	3	2	1	0	1	2	3
SBP (mmHg)	<91	91-100	101-110	111-219			≥220
HR (beats/min)	<41		41-50	51-90	91-110	111-130	≥131
RR (cycles/min)	<9		9-11	12-20		21-24	≥25
*T* (°C)	<35.1		35.1-36	36.1–38	38.1-39	≥39.1	
SaO_2_ (%)	<92	92-93	94-95	≥96			
Oxygen support		Yes		No			
AVPU				A			V, P, or U

**(d):** 

mREMS							
Variable	0	1	2	3	4	5	6
Age (years)	<45	45-64		65-74	≥75		
SBP (mmHg)		90-109	80-89		<80		
	110-159	160-199	≥200	130-159			
HR (beats/min)			55-69	40-54	<40		
	70-109		110-139	140-179	≥180		
RR (cycles/min)		10-11	6-9		<6		
	12-24	25-34		35-49	≥50		
SaO_2_ (%)	≥90	86-89		75-85	<75		
GCS	14 or 15		8-13			5-7	3 or 4

**(e):** 

RTS							
Variable	0	1	2	3	4		
SBP (mmHg)	0	1-49	50-75	76-89	≥90		
RR (cycles/min)	0	1-5	6-9	≥30	10-29		
GCS	3	4-5	6-8	9-12	13-15		

RTS = 0.9368 GCS + 0.7326 SBP + 0.2908 RR. The mREMS used in this study was modified from the traditional REMS [47] to achieve better prediction performance for the trauma population [6].

**Table 2:** Characteristics of the survival and nonsurvival groups among patients with multiple trauma admitted during the daytime and nighttime.

	Daytime			Nighttime		
	Survival	Nonsurvival	*p* value	Survival	Nonsurvival	*p* value
*n*	917	153		651	97	
Female *n* (%)	323 (35.2)	48 (31.4)	0.404	183 (28.1)	15 (15.5)	0.012
Age (years)	54 [44, 67]	54 [42, 68]	0.885	49 [38, 59]	45 [36, 56]	0.295
LOS (days)	9 [4, 15]	1 [0, 5]	<0.001	8 [1, 14]	1 [0, 3]	<0.001
*T* (°C)	37.0 [36.7, 37.0]	36.5 [36.0, 37.0]	<0.001	37.0 [36.7, 37.0]	36.2 [35.6, 37.0]	<0.001
HR (beats/min)	80 [75, 88]	85 [65, 115]	0.139	80 [75, 88]	97.5 [76, 125]	<0.001
RR (cycles/min)	20 [18, 20]	22 [20, 30]	<0.001	20 [18, 21]	26.5 [20, 31]	<0.001
SBP (mmHg)	134 [124, 147]	131 [93, 163]	0.209	132 [120, 144]	124 [95, 156]	0.036
SaO_2_ (%)	98 [97, 98]	95 [87, 98]	<0.001	98 [97, 99]	91 [82, 97]	<0.001
AVPU	0 [0, 0]	3 [2, 3]	<0.001	0 [0, 0]	3 [2, 3]	<0.001
GCS	15 [15, 15]	3 [3, 7]	<0.001	15 [15, 15]	3 [3, 8]	<0.001
Trauma mechanism *n* (%)			<0.001			0.001
Traffic accident	427 (46.6)	86 (56.2)		340 (52.2)	60 (61.9)	
High fall	108 (11.8)	28 (18.3)		53 (8.1)	17 (17.5)	
Crushing injury	21 (2.3)	11 (7.2)		15 (2.3)	3 (3.1)	
Cut/pierce	9 (1.0)	3 (2.0)		16 (2.5)	4 (4.1)	
Burn	8 (0.9)	0 (0.0)		5 (0.8)	1 (1.0)	
Tumble injury	315 (34.4)	16 (10.5)		191 (29.3)	9 (9.3)	
Struck	29 (3.2)	9 (5.9)		31 (4.8)	3 (3.1)	
Score of triage tool						
NEWS	2 [2, 4]	10 [6, 12]	<0.001	2 [2, 4]	11 [8, 14]	<0.001
MEWS	1 [1, 2]	5 [4, 7]	<0.001	1 [1, 2]	5 [4, 8]	<0.001
SEWS	0 [0, 1]	5 [3, 8]	<0.001	0 [0, 1]	6 [3, 8]	<0.001
mREMS	4 [2, 5]	10 [8, 13]	<0.001	3 [1, 4]	11 [7, 13]	<0.001
RTS	7.8 [7.8, 7.8]	5.0 [4.1, 6.0]	<0.001	7.8 [7.8, 7.8]	4.7 [4.1, 6.9]	<0.001

**Table 3:** Characteristics of the minor and severe trauma groups among patients with multiple trauma admitted during the daytime and nighttime.

	Daytime			Nighttime		
	Minor trauma	Severe trauma	*p* value	Minor trauma	Severe trauma	*p* value
*n*	703	367		495	253	
Female *n* (%)	263 (37.4)	108 (29.4)	0.011	149 (30.1)	49 (19.4)	0.002
Age (years)	54 [44, 68]	53 [45, 66]	0.403	49 [38, 60]	47 [38, 56]	0.188
LOS (days)	8 [1, 13]	8 [1, 19]	0.008	6 [0, 11]	8 [1, 18]	0.001
*T* (°C)	37.0 [36.7, 37.0]	36.8 [36.5, 37.0]	0.087	37.0 [36.7, 37.0]	36.8 [36.3, 37.0]	<0.001
HR (beats/min)	80 [75, 88]	82 [72, 95]	0.032	80 [75, 88]	86 [78, 101]	<0.001
RR (cycles/min)	20 [18, 20]	20 [18, 22]	<0.001	20 [18, 20]	20 [20, 25]	<0.001
SBP (mmHg)	132 [125, 146]	135 [116, 153]	0.315	133 [123, 144]	126.5 [107, 143]	<0.001
SaO_2 (%)	98 [97, 98]	97 [95, 98]	<0.001	98 [97, 99]	97 [92, 98]	<0.001
AVPU	0 [0, 0]	1 [0, 2]	<0.001	0 [0, 0]	1 [0, 2]	<0.001
GCS	15 [15, 15]	13 [4, 15]	<0.001	15 [15, 15]	13 [4, 15]	<0.001
Trauma mechanism *n* (%)			<0.001			<0.001
Traffic accident	318 (45.2)	195 (53.1)		249 (50.3)	151 (59.7)	
High fall	65 (9.2)	71 (19.3)		30 (6.1)	40 (15.8)	
Crushing injury	10 (1.4)	22 (6.0)		6 (1.2)	12 (4.7)	
Cut/pierce	8 (1.1)	4 (1.1)		14 (2.8)	6 (2.4)	
Burn	6 (0.9)	2 (0.5)		3 (0.6)	3 (1.2)	
Tumble injury	274 (39.0)	57 (15.5)		170 (34.3)	30 (11.9)	
Struck	22 (3.1)	16 (4.4)		23 (4.6)	11 (4.3)	
Score of triage tool						
NEWS	2 [2, 4]	5 [3, 9]	<0.001	2 [2, 4]	5 [3, 10]	<0.001
MEWS	1 [1, 2]	2 [1, 5]	<0.001	1 [1, 2]	2 [1, 4]	<0.001
SEWS	0 [0, 1]	1 [0, 5]	<0.001	0 [0, 1]	1 [0, 4]	<0.001
mREMS	4 [2, 5]	6 [4, 10]	<0.001	3 [1, 4]	4 [2, 8]	<0.001
RTS	7.8 [7.8, 7.8]	7.8 [5.0, 7.8]	<0.001	7.8 [7.8, 7.8]	7.8 [6.0, 7.8]	<0.001

**Table 4:** Comparison of AUROCs, optimal cut-offs, sensitivity, and specificity for identifying in-hospital mortality.

Score	Daytime					Nighttime					*p* value
	AUROC	95CI	Opt cut-off	Sen	Sp	AUROC	95CI	Opt cut-off	Sen	Sp	
MEWS	0.95	0.93–0.97	>2	0.9	0.89	0.93	0.9–0.96	>3	0.86	0.94	0.384
NEWS	0.95	0.93–0.97	>4	0.94	0.82	0.94	0.92–0.97	>5	0.9	0.89	0.708
SEWS	0.95	0.93–0.97	>2	0.84	0.93	0.94	0.91–0.97	>2	0.9	0.92	0.683
mREMS	0.94	0.92–0.97	>7	0.83	0.94	0.92	0.88–0.96	>7	0.79	0.95	0.286
RTS	0.93	0.9–0.95	<7.68	0.9	0.9	0.93	0.9–0.97	<7.00	0.88	0.92	0.87

**Table 5:** Comparison of AUROCs, optimal cut-offs, sensitivity, and specificity for identifying severe trauma.

Score	Daytime					Nighttime					*p* value
	AUROC	95CI	Opt cut-off	Sen	Sp	AUROC	95CI	Opt cut-off	Sen	Sp	
MEWS	0.78	0.75–0.81	>2	0.53	0.94	0.78	0.75–0.82	>2	0.53	0.93	0.95
NEWS	0.8	0.77–0.83	>4	0.62	0.89	0.8	0.76–0.83	>4	0.65	0.85	0.885
SEWS	0.78	0.76–0.81	>1	0.55	0.92	0.78	0.74–0.81	>1	0.55	0.92	0.818
mREMS	0.75	0.72–0.78	>7	0.44	0.98	0.69	0.65–0.73	>7	0.37	0.97	0.019
RTS	0.75	0.73–0.78	<7.18	0.52	0.97	0.74	0.71–0.78	<7.68	0.52	0.95	0.619

## Data Availability

The datasets used and/or analyzed during the current study are available from the corresponding author on reasonable request.
